The article "Effects of Personalized Nursing plus Dietary Nursing Management on LP-PLA2, Hcy Levels, and Quality of Life in Elderly Patients with Acute Coronary Syndrome" was retracted in 2023. Reasons: unreliable results or conclusions; concerns about the data; concerns about the peer review; concerns about the citations.

# Effects of Personalized Nursing plus Dietary Nursing Management on LP-PLA2, Hcy Levels, and Quality of Life in Elderly Patients with Acute Coronary Syndrome

**DOI:** 10.1155/2022/8770996

**Published:** 2022-08-17

**Authors:** Fan Luo, Jingrui Qi, Li Zhao, Yu Wang, Mei Yang

**Affiliations:** ^1^Department of Geratology, Cangzhou Central Hospital, Cangzhou, China; ^2^Department III of Ultrasound, Cangzhou Central Hospital, Cangzhou, China

## Abstract

**Objective:**

To explore the effect of individual nursing combined with dietary management on blood glucose levels and quality of life in elderly patients with acute coronary syndrome with diabetes.

**Method:**

This study included 68 elderly patients who underwent acute coronary syndrome at Department of Emergency in our hospital from January 2018 to January 2020. And they were assigned to a control group (*n* = 34) treated with individual nursing and a research group (*n* = 34) treated with individual nursing and dietary management according to the random number table. A comparison of the changes in blood glucose levels, anxiety and depression, quality of life, and nursing satisfaction was made between groups before and after nursing.

**Result:**

Before nursing, the differences in blood glucose levels, SAS scores, and SDS scores between groups were not considered statistically significant (*P* > 0.05). After nursing, the blood glucose levels, SAS, and SDS levels of patients in both groups significantly decreased, and the research group presented a higher decrease when compared with the control group (*P* < 0.05). The short form health survey (SF-36) showed that the research group had higher scores in physical function (PF), general health (GH), vitality (VT), mental health (MH), social function (SF), role-physical (RP), bodily pain (BP), and role-emotional (RE) compared with the control group (*P* < 0.05). The satisfaction survey presented that the research group had a significantly higher total score than the control group [(91.40 ± 5.23) vs. (86.61 ± 7.14), *P* < 0.05].

**Conclusion:**

The combination of individual nursing and dietary management not only effectively reduces glycosylated hemoglobin levels and anxiety and depression but also wins better nursing satisfaction in the treatment of acute coronary syndrome in elderly patients. Moreover, their quality of life has been significantly improved after discharge.

## 1. Introduction

Acute coronary syndrome (ACS) usually results from sudden rupture or erosion of plaque inside the coronary artery that leads to thrombus and acute stenosis or blockage. It is common among the elderly and the main reason for death and disability caused by coronary heart disease [1]. Sympathetic excitation, increased blood viscosity, and increased myocardial oxygen consumption lead to rupture or erosion of unstable atherosclerotic plaques, causing platelet agglutination and consequent thrombosis, which can eventually result in acute or subacute myocardial hypoxia or ischemia, or even myocardial injury [2]. Coronary heart disease is often accompanied by multiple complications, among which patients with type 2 diabetes mellitus account for about 20%–30%. Dyslipidemia can exist in patients with coronary heart disease and type 2 diabetes. When the two diseases interact, disorders of lipid metabolism are more severe, while blood glucose levels have pathogenic mechanisms that lead to vascular atherosclerosis, and their levels are sensitive to the vascular condition and are of great value for prediction, diagnosis, and prognostic assessment [3, 4].

It is challenging to standardize diagnosis and treatment, improve the successful treatment rate, and improve the quality of life and long-term survival rate in the treatment of ACS with diabetes with the acceleration of population aging in China. Individualized care is patient-centered and places greater emphasis on primary care. Previous studies have shown that individualized nursing interventions are effective in improving the quality of life of patients, combined with the importance of diet in elderly patients with acute coronary syndrome combined with diabetes. The aim of this study was to investigate the effect of individualized care combined with dietary management on postoperative glycated hemoglobin levels and quality of life in elderly patients with ACS combined with diabetes mellitus, with a view to clinical reference.

## 2. Subjects and Methods

### 2.1. Research Subjects

Sixty-eight elderly patients with ACS combined with diabetes mellitus attending our emergency department from January 2018 to January 2020 were included in this study for prospective analysis, and all patients in this study were divided into a control group (*n* = 34) and a study group (*n* = 34). The ethics committee of our hospital approved this study.

### 2.2. Inclusion and Exclusion Criteria

#### 2.2.1. Inclusion Criteria

1. Patients who met the standards in guidelines for emergency rapid diagnosis and treatment of acute coronary syndrome, and whose diagnosis was confirmed by electrocardiogram and relevant laboratory tests [5];
2. Clinically diagnosed as diabetes;
3. Patients with age ≥ 60 years old;
4. Patients who experienced percutaneous coronary intervention, including balloon angioplasty, and stent implantation;
5. Patients with a normal mentality and the ability to communicate;
6. Patients who had been informed and voluntarily participated in this study

#### 2.2.2. Exclusion Criteria

1. Patients who were retired medical staffs;
2. Patients with malignant tumors;
3. Patients with liver and kidney dysfunction;
4. Patients with ACS followed by thyroid dysfunction and leukemia.

### 2.3. Nursing Methods

#### 2.3.1. Control Group

The control group was provided with individual nursing.

1. Medication guidance: medical staffs gave the prescriptions with mild adverse reactions and low cost based on the conditions of patients, relevant laboratory tests, drug contraindications, history of drug allergy, financial status, etc. Next, they instruct patients to take the medication and monitor the efficacy and side effects in real time. If patients experience serious adverse reactions, medical staff should immediately inform the physician in order to adjust the dose and improve patient compliance.
2. Psychological intervention: medical staffs provided specific psychological counseling after communicating many times. Provided that patients were not confident about treatment, medical staffs shared successful cases to enhance their confidence. If patients refused treatment because of costly expenses, medical staffs helped raise medical expenses through crowdfunding, and donations. In addition, medical staffs explained the conditions of patients and their required nursing in simple words to facilitate their understanding and ease their anxiety, thereby building a good nurse-patient relationship.
3. Health education: medical staffs threw lectures to analyze the causes, clinical manifestations, and treatment of ACS and instruct patients to have such good habits as normal rest, proper exercise, smoking cessation and quitting alcohol, and a scientific diet.
4. Discharge guidance: when patients left the hospital, they were reminded to take medications as prescribed by physicians. (4) Family members assume supervisory responsibility to help patients maintain good lifestyle habits, for example, patients perform daily exercises such as jogging, tai chi and bada-jen, drink tea appropriately, take adequate fiber, and patients must seek medical advice if they are unwell. Medical staff follows up with discharged patients from time to time through WeChat, phone calls, and SMS to understand their condition and answer their questions, for 12 months per patient.

#### 2.3.2. Research Group

The research group was provided with dietary management plus the same individual nursing as the control group. Specific steps for dietary management are as follows:

1. First was to evaluate the daily diet of patients to establish a record.
2. The second was to collect and record general information like height, weight, work, blood pressure, and blood sugar,. Then, based on the dietary preferences of patients, medical staffs drew a calorie chart and designed a scientific and reasonable recipe [6]. In addition to rice and flour, patients also eat whole grains such as sweet potatoes, purple potatoes, corn, potatoes, yams, buckwheat, and oatmeal to meet their calorie needs. They also eat fresh vegetables and seasonal fruit every day for vitamins, and appropriate amounts of meat, eggs, milk, and soya products for protein.
3. Trained medical staffs instructed families to cook meals by recipes.
4. After discharge, patients were requested to regularly follow the recipe to have a healthy diet. In the meantime, patients appropriately drank weak tea instead of strong tea, were forbidden to have tea with drugs or at night, and monitored blood pressure and blood sugar daily.

### 2.4. Observation Indexes

1. The changes in glycosylated hemoglobin levels before and after nursing (at discharge) were compared between the two groups. Before and after the intervention, the fasting blood in the morning was collected and the glycosylated hemoglobin level was measured by the hospital's automatic biochemical analyzer (Jinan Oulaibo Scientific Instrument Co., Ltd.; bk-200). The normal value of glycosylated hemoglobin is 4%∼6%.
2. Assessed the anxiety and depression of the two groups with the self-rating anxiety scale (SAS) [7] and self-rating depression (SDS) before and after nursing [8].
3. Assessed the quality of life of the two groups with short-form health survey 36 (SF-36), after follow-up, consisting of eight aspects like physical function (PF), general health (GH), vitality (VT), mental health (MH), social function (SF), role-physical function (RP), bodily pain (BP), and role-emotional function (RE), with a total of 36 items [9].
4. Created a nursing satisfaction questionnaire that consisted of nursing attitude, health education, humanistic care, nursing efficacy, and discharge guidance, with 20 points for each item and a total score of 100 points. A higher score meant better satisfaction, and this collection was completed within one week after discharge.

### 2.5. Statistical Analysis

In this study, the data was analyzed using SPSS23.0. The enumeration data were expressed as *n* (%) using the Chi-square test, and the measurement data were expressed as the mean ± standard deviation and compared between groups using *t*-test. *P* < 0.05 implied a statistical significance.

## 3. Results

### 3.1. Comparison of General Data

There were 34 patients in each group, and there was no significant difference in gender, age, clinical classification, hypertension, and other general data (*P* > 0.05), as shown in Table 1.

### 3.2. Comparison of Glycosylated Hemoglobin Levels between Groups before and after Nursing

There was no significant difference in the level of glycosylated hemoglobin between the two groups before nursing (*P* > 0.05). After nursing, the level of glycosylated hemoglobin decreased significantly (*P* < 0.001), and the level of glycosylated hemoglobin in the study group was significantly lower than that in the control group (*P* < 0.05), as shown in Table 2.

### 3.3. Comparison of SAS and SDS Scores before and after Nursing

No significant difference was observed in SAS and SDS scores between groups before nursing (*P* > 0.05). After nursing, the SAS and SDS scores of the two groups both significantly decreased, and the research group had lower SAS and SDS scores when compared with the control group (*P* < 0.05). See Table 3.

### 3.4. Comparison of SF-36 Scores after Follow-Up

The SF-36 score showed that the research group had higher scores in PF, GH, TV, MH, SF, RP, BP, and RE when compared with the control group (*P* < 0.05). See Table 4, and Figure 1.

### 3.5. Comparison of Nursing Satisfaction after Follow-Up

The satisfaction survey showed that patients in the research group gave higher total scores than patients in the control group, and they gave higher scores in nursing efficacy and discharge guidance (*P* < 0.05). See Table 5.

## 4. Discussion

ACS is a common and serious cardiovascular disease seen in the elderly, postmenopausal women, and people with a history of smoking, hypertension, diabetes, hyperlipidemia and abdominal obesity, and a family history of early coronary heart disease [10]. It presents with paroxysmal chest pain and tightness, leading to arrhythmias, heart failure, and even sudden death, thus, affecting the quality of life and life expectancy [11, 12].

Compared with other traditional risk factors, glycosylated hemoglobin reflects vascular conditions more sensitively. Their levels are positively correlated with the occurrence of cardiovascular malignant diseases and mortality. The increase in glycated hemoglobin induces vascular inflammation and promotes the formation and rupture of arterial plaque, which leads to various cardiovascular diseases. Studies have found that acute cardiovascular disease is closely related to plaque stability, and if plaque is in an unstable state, it can lead to increased blood glucose and patients are more likely to develop malignant cardiovascular disease [13]. The increase in glycosylated hemoglobin brings damage to blood vessels, leading to coronary artery disease, peripheral vascular disease, cerebrovascular disease, and venous thrombosis. The local thrombus is gradually replaced by fibrous tissue, with changes in smooth muscle proliferation in the process, thereby increasing the risk of cardiac, cerebral, and peripheral vascular atherosclerosis, ultimately leading to a greatly increased risk of myocardial infarction and stroke [14, 15].

Individual nursing meets the physiological, psychological, social, and spiritual needs of patients with ACS with diabetes and improves their prognosis. Individual nursing is patient-centered, emphasizes primary nursing, and provides more satisfying comprehensive nursing. Individualized nursing interventions are used to alleviate patients' dysphoria, increase their awareness of the disease, and play a positive role in strengthening their immune system and creating a good therapeutic environment [16]. Poor diet directly worsens the patient's condition. If patients consume too much fat, sodium, and sugar, it can directly lead to increased blood pressure, blood sugar and lipids, metabolic disorders, and elevated Lp-PLA2 and Hcy levels. It is therefore necessary to develop scientific dietary recipes to correct metabolic disorders [17, 18].

In this study, the decrease in glycosylated hemoglobin levels was significantly lower in the study group than in the control group aftercare, and SAS and SDS scores were lower in the study group, suggesting that individualized care combined with dietary management provides not only specific nursing interventions, especially in physical and psychological aspects but also detailed medication instructions. Psychological intervention is to relieve their anxiety and depression, deliver health education and enhance self-confidence, and specific dietary management is to improve their diets and nutritional balance. In addition, discharge instructions are a solution to their postdischarge worries. In the treatment of ACS combined with diabetes mellitus, there is a certain damage to the body of elderly patients, and with various physical functions declining with age, they are prone to a series of adverse reactions, and most patients experience adverse reactions followed by poor mood, which affects the efficacy and reduces the quality of life [19, 20].

In China, the current focus of our medical service is to improve the quality of life, including the conditions of patients and their survival. This study found that after follow-up, the research group had a better quality of life compared with the control group, and also gives better nursing satisfaction. Most elderly patients experience ACS with diabetes because of smoking, hypertension, diabetes, hyperlipidemia, and abdominal obesity. Individualized care provides patients with targeted care strategies and effective dietary management to help them manage their blood glucose and intervene [21]. Proper dietary management is essential for self-management in patients with chronic diseases, and most elderly ACS patients with diabetes have difficulty matching their daily diet due to low education, low health awareness, and financial constraints. However, in this study, patients were provided with tailor-made recipes and taught cooking skills by medical staff in person to help patients eat scientifically and with strict control of daily intake by patients, which helps to reduce cardiac load and regulate metabolic disturbances. Eating more coarse fiber food has four benefits. Firstly, it promotes bowel movement, improves gastrointestinal function, and prevents constipation and even bowel cancer. The second is to improve blood sugar response and lower postmeal blood sugar to treat diabetes. The third is to reduce the cholesterol in plasma to prevent and treat hyperlipidemia and cardiovascular disease. The fourth is to control weight so as to reduce the occurrence of obesity [22, 23]. In the meantime, it is also recommended to appropriately drink tea because of its role in anticoagulation and promoting fibrinolysis. Tea polyphenols can improve the permeability of microvascular walls, effectively enhancing the elasticity and resistance of myocardial and vascular walls and reducing the severity of atherosclerosis [24]. Moreover, caffeine and theophylline directly excite the heart, expand coronary arteries, and enhance myocardial function. In this study, the baseline data of SF-36 in the two groups were not collected, which may weaken the research conclusion of this study. However, since the two groups of patients were randomly grouped through the random number table, it is reasonable to believe that the baseline levels of SF-36 in the two groups are similar.

Non-ST-segment elevation coronary syndromes are usually treated with antimyocardial ischemic drugs to reduce myocardial oxygen consumption, dilate coronary arteries, increase coronary blood flow and relieve myocardial ischemia [25]. *β*-receptor antagonists can reduce myocardial oxygen consumption, reduce recurrent episodes of myocardial ischemia, and may improve patient prognosis [26]. Calcium channel blockers are the first choice for vasospastic angina and can also be used in patients whose symptoms are not controlled despite adequate nitrate and beta antagonist therapy [27]. Antiplatelet therapy is primarily an antiplatelet coagulation therapy to prevent thrombosis [28].

There is no evidence-based treatment for this disease, but some TCM treatments or medications can relieve symptoms. The clinical manifestations of ACS are breath power deficiency, Yang deficiency, Yin deficiency, and breath power-Yin deficiency or breath power -Yang deficiency, as well as breath power stagnation, blood stasis, phlegm blockage and cold condensation, and blood stasis is a prevalent pathological feature [29]. The blood-activating herbs Radix Paeoniae, *Salviae miltiorrhiza*, Rhizoma Chuanxiong, *Panax notoginseng*, peach kernel, and rhubarb in wine have certain plaque-stabilizing effects, and their plaque-stabilizing effects vary [30]. Rhubarb made from blood-breaking herbal wine has the best plaque-stabilizing effect, almost similar to that of the western drug simvastatin, followed by *Panax notoginseng* [31]. The mechanism may be related to the regulation of lipid metabolism and the inhibition of inflammatory responses, but there may be differences in the link and intensity of action [30–32].

## 5. Conclusion

In conclusion, the combination of individual nursing and dietary management not only effectively reduces glycosylated hemoglobin levels and relieves anxiety and depression, but also wins higher nursing satisfaction in the treatment of acute coronary syndrome in elderly patients. Moreover, their quality of life has been significantly improved after discharge. There is some geographical variation in this study, the patients in the study may not be representative of the entire affected population, and secondly, there may be some methodological heterogeneity and clinical heterogeneity. In conclusion, we need a more detailed experimental design for clinical studies.

## Figures and Tables

**Figure 1:** Comparison of quality of life scores between the two groups.

**Table 1:** Comparison of general data [*n* (%), ($\bar{x}\pm s$)].

Group	*n*	Gender		Age	Type		Hypertension
		Male	Female		Acute myocardial infarction	Unstable angina	
Control group	34	21	13	68.21 ± 9.47	18	16	29
Research group	34	23	11	69.58 ± 9.54	20	14	30
*t*		0.258		0.594	0.239		0.128
*P*		0.400		0.554	0.404		0.500

**Table 2:** Comparison of glycosylated hemoglobin between groups before and after nursing ($\bar{x}\pm s$).

Group	*n*	Before nursing	After nursing	*t*	*P*
Control group	34	10.08 ± 1.46	6.65 ± 1.35	10.058	<0.001
Research group	34	9.93 ± 1.57	6.01 ± 0.96	12.421	<0.001
*t*		0.408	2.253		
*P*		0.684	0.028		

**Table 3:** Comparison of SAS and SDS scores before and after nursing ($\bar{x}\pm s$).

Group	*n*	SAS		SDS	
		Before nursing	Before nursing	Before nursing	After nursing
Control group	34	65.39 ± 7.27	49.22 ± 5.51^*∗*^	29.14 ± 3.45	19.12 ± 2.47^*∗*^
Research group	34	66.67 ± 7.45	38.47 ± 4.32^*∗*^	28.98 ± 3.13	14.28 ± 1.79^*∗*^
*t*		0.717	8.953	0.200	9.252
*P*		0.476	<0.001	0.842	<0.001

*Note.* Comparison with before nursing, (^*∗*^*P* < 0.05).

**Table 4:** Comparison of SF-36 scores after follow-up ($\bar{x}\pm s$).

Item	Control group	Research group	*t*	*P*
PF	86.14 ± 5.98	95.78 ± 4.51	7.505	<0.001
GH	42.21 ± 7.99	81.03 ± 1.95	27.520	<0.001
TV	55.78 ± 6.91	93.26 ± 3.37	28.430	<0.001
MH	66.82 ± 7.56	88.67 ± 3.56	15.250	<0.001
SF	87.69 ± 8.57	104.41 ± 9.77	7.502	<0.001
RP	85.48 ± 17.92	94.16 ± 8.78	2.536	0.014
BP	60.72 ± 6.53	71.87 ± 10.13	5.394	<0.001
RE	51.42 ± 5.34	89.45 ± 6.74	25.790	<0.001

**Table 5:** Comparison of nursing satisfaction ($\bar{x}\pm s$).

Type	Control group (*n* = 34)	Research group (*n* = 34)	*t*	*P*
Nursing attitude	17.75 ± 1.34	18.01 ± 1.12	0.868	0.388
Health education	17.46 ± 1.01	17.89 ± 1.24	1.568	0.122
Humanistic care	18.13 ± 1.04	18.36 ± 0.87	0.989	0.326
Nursing efficacy	16.84 ± 2.23	18.98 ± 0.51	5.455	<0.001
Discharge guidance	16.43 ± 2.51	18.16 ± 1.32	3.557	<0.001
Total score	86.61 ± 7.14	91.40 ± 5.23	3.156	0.002

## Data Availability

The datasets used during the present study are available from the corresponding author upon reasonable request.
